The article "Analysis of Coronary Artery Lesion Degree and Related Risk Factors in Patients with Coronary Heart Disease Based on Computer-Aided Diagnosis of Coronary Angiography" was retracted in 2023. Reasons: unreliable results or conclusions; lack of ethics approval or compliance; concerns about the data; concerns about the peer review.

# Analysis of Coronary Artery Lesion Degree and Related Risk Factors in Patients with Coronary Heart Disease Based on Computer-Aided Diagnosis of Coronary Angiography

**DOI:** 10.1155/2021/2370496

**Published:** 2021-12-14

**Authors:** Xuan Wang, Dehao Yu, Junrui Wang, Junjie Huang, Wenqing Li

**Affiliations:** ^1^Department of Cardiology, Juye County People's Hospital, Heze, 274900 Shandong, China; ^2^Department of Rehabilitation Medicine, Neck, Shoulder and Back Pain Treatment, Hospital of Shandong Provincial Medical Sciences Academy, Jinan, 250014 Shandong, China; ^3^Department of Neurology, Juye County People's Hospital, Heze, 274900 Shandong, China; ^4^Department of Haematology, Juye County People's Hospital, Heze, 274900 Shandong, China; ^5^Department of Endocrinology, Juye County People's Hospital, Heze, 274900 Shandong, China

## Abstract

A combination of various risk factors results in the development of coronary heart disease. The earlier that one identifies and deals with reversible risk factors for coronary heart disease, the greater the chance of recovery. The main goal of this research is to learn whether risk variables are associated with greater extent of coronary artery disease in people with coronary heart disease. This article selects 290 patients who had had coronary angiography in our hospital from September 2018 to March 2019 using a retrospective research and analytic methodology. Coronary angiography split the patients into two groups: those with coronary heart disease and those without. To determine the correlation between risk factors and a score related to heart disease, computer-aided statistical analysis of data about the differences in those risk factors was performed. The results were analyzed using the Spearman correlation and partial correlation, and the relationship between risk factors and Gensini score was analyzed by multiple linear regression. For the analysis, binary logistic regression was used to calculate the correlation between the risk factors of coronary heart disease and the probability of developing coronary heart disease. The findings concluded that increased age, smoking, elevated hs-CRP, HbA1c, hypertension, diabetes, and hyperuricemia are all contributors to coronary heart disease. Coronary heart disease is an independent risk factor for this condition. Many of the factors that play a role in the long-term development of the severity of coronary artery disease, such as hypertension, diabetes, smoking, elevated hs-CRP, decreased HDL-C, raised LDL-C, and TG, are commonly found in men. hs-CRP is the primary risk factor for the degree of coronary artery stenosis and could contribute to the progression of the condition by playing a major role in creating more stenosis.

## 1. Introduction

Cardiovascular disease as shown in Figure 1 is one of the important threats to human health currently. Worldwide, the annual mortality of 1/3 of the entire population can be attributed to this sickness. According to this information, the greatest proportion of cardiovascular disease mortality was due to coronary heart disease. In 1990, almost 35% more people died from coronary heart disease (CHD) than in 1990. In 2015, about 110 million people were impacted by coronary heart disease, resulting in 8.9 million fatalities. One of the leading causes of death around the world has become this. Despite being less common in Europe and the US, the incidence and death of coronary heart disease in my nation have been rising quickly over the past three decades. Coronary atherosclerosis is the root cause of coronary heart disease. Coronary atherosclerosis incidence is rising due to improvements in people's living standards and changes in dietary patterns. It was formerly thought of to be a degenerative disease, since atherosclerotic plaque is manifested as a buildup of lipids and necrotic tissue [1–6].

A landmark study known as the Framingham Heart Study initially laid out the notion of “risk factors” in 1961. The repeatedly proposed risk factors for coronary heart disease were derived from a considerable amount of clinical research in other countries. To date, at least 300 important risk factors for coronary heart disease have been discovered. So far, coronary heart disease is considered to be caused by both hereditary and environmental risk factors working together to make someone more susceptible to developing it. Cumulative research has demonstrated that established risk factors for coronary heart disease, such as age, gender, dyslipidemia, hypertension, diabetes, and smoking, all contribute to a person's likelihood of developing the condition. It is also necessary to look at other risk factors, such as hyperuricemia, inflammation, obesity, and psychosocial variables, which are significantly connected to coronary heart disease. The other risk factors are unpredictable (including age and gender). However, we can overcome those uncontrollable risk factors through artificial control. The earlier that one identifies and deals with reversible risk factors for coronary heart disease, the greater the chance of recovery. Although cardiovascular illnesses are the third leading cause of death, researchers have found that the vast majority may be averted by managing risk factors, such as exercise, a proper diet, treatment of high blood pressure, a healthy weight, and cessation of smoking. More than 80% of coronary heart disease can be prevented by the removal of risk factors such as obesity, bad diet, and lack of exercise [7–11].

Although people's lifestyles and eating habits have changed in recent years, as my country has steadily entered an aging culture, the incidence of coronary heart disease has been increasing year by year. Although age does contribute to the risk of developing coronary heart disease and the degree of coronary stenosis, evidence collected from clinical studies shows that the incidence of coronary heart disease and the degree of coronary stenosis rise with age [12]. Although there are several risk factors for coronary heart disease, such as genetics, smoking, and diet, age is one of the uncontrollable ones. As age increases, the coronary artery intima and media fibrosis increase, resulting in greater extracellular matrix deposition, a decrease in endothelial cell density, and the presence of more multinucleated endothelial cells, which all contribute to endothelial cell failure. The impact of numerous risk factors on the artery wall increases with age.

Coronary angiography, as an invasive examination method, mainly fills the coronary lumen with a contrast agent to reflect the condition of coronary artery stenosis. It is currently the most common method for diagnosing coronary artery disease and guiding treatment options. The Judkins method is often used to puncture the femoral artery or radial artery, and the left main trunk, left anterior descending artery, circumflex artery, and right coronary artery are observed in multiple positions. The angiography revealed that the blood vessels with diameter ≥ 1.5 mm and stenosis≥50% were meaningful lesions. The Gensini scoring system [13] divides the coronary arteries into 15 segments and formulates different weighting coefficients according to different segments of the diseased blood vessel. Considering the number, location, and stenosis of coronary artery disease, it is a very effective method to assess the degree of coronary artery disease, and it is also one of the most commonly used clinical methods. The more severe the coronary artery disease, the higher the Gensini score. Gensini scores are currently widely used in clinical trials.

This study is aimed at examining the relationship between coronary artery disease risk factors and the level of coronary artery disease in patients with coronary artery disease based on computer-assisted technology and will use the Gensini score as a means of measuring this. Clinical judgment of the complexity of coronary heart disease was strengthened by providing fresh evidence.

## 2. Related Work

Studies abroad had shown that hypertension played a very important role in the occurrence and development of coronary heart disease and was one of the main risk factors for coronary heart disease [14]. Hypertension could accelerate the formation of atherosclerosis and increase the risk of coronary heart disease by 2 to 3 times. In a meta-analysis involving 1 million people [15], blood pressure fluctuations in patients were closely related to the mortality rate of coronary heart disease, with fluctuations ranging from 115/75 mmHg to 185/115 mmHg. They found that every 20 mmHg increase in systolic blood pressure (or every 10 mmHg increase in diastolic blood pressure) doubled the risk of fatal coronary events. Hypertension could lead to an increase in coronary perfusion pressure and vascular wall tension. Continuously increased tension could cause damage to the vascular intima, lipid deposition, and smooth muscle hyperplasia and finally the formation of atherosclerotic plaques. In addition, the mechanical pressure of hypertension on the coronary artery wall increased, and the vascular endothelium was prone to damage, releasing endothelin-1 and other vasoactive substances, causing vasoconstriction. At the same time, under the action of chemical mediators caused by inflammation, the blood vessel wall became thick and stiff. The formation of coronary atherosclerotic plaque and a variety of risk factors caused coronary artery stenosis.

Blood glucose played an important role in the process of coronary artery disease, but it is easily affected by many factors, such as diet, and fluctuates greatly. Glycated hemoglobin was one of the most easily detected biomarkers in diabetic patients. It was the product of the nonenzymatic glycation reaction of hemoglobin in the blood under the action of hyperglycemia, and its main form is HbA1c. Farrag et al. [16] found that in patients with coronary heart disease with diabetes, HbA1c level could predict the degree of coronary artery disease. A systematic analysis of the global burden of disease [17] showed that from 1990 to 2015, smoking caused more than 5 million deaths each year. The US Centers for Disease Control and Prevention reported [18] that the life expectancy of male and female smokers would be shortened by an average of 13.2 and 14.5 years, respectively. Nyboe et al. found [19] that smoking could aggravate the severity of coronary heart disease to a certain extent. There was a certain correlation between smoking and coronary artery disease in patients with coronary heart disease. Smoking could cause changes in the structure of vascular endothelial cells, and endothelial damage was considered to be the initiating factor of atherosclerosis [20]. Long-term smoking would reduce coronary endothelial cell-dependent vasodilation, increase platelet aggregation and increase fibrinogen, and increased the level of inflammatory factors, causing and aggravating the formation of atherosclerotic plaques.

Previous studies had shown [21–23] that abnormal blood lipid metabolism was closely related to coronary atherosclerosis, and elevated blood lipid levels (except HDL-C) could increase the risk of coronary heart disease. Xiao et al. confirmed [24] that the increase of total cholesterol (TC) and low-density lipoprotein cholesterol (LDL-C) and the decrease of high-density lipoprotein (HDL-C) are one of the most important independent risk factors for coronary heart disease. Malley et al. [25] also found that lipid-lowering therapy has significant benefits in reducing coronary heart disease events. The PROCAM study [26] suggested that cholesterol absorption efficiency was positively correlated with the risk of coronary events, and regardless of the LDL level, the lower the HDL level, the greater the risk of coronary heart disease.

Epidemiological investigation [27] showed that patients with hyperuricemia were closely related to coronary heart disease, but the exact mechanism of hyperuricemia inducing coronary heart disease was not yet fully understood. Hyperuricemia was a disorder of purine metabolism, and its incidence had been increasing in recent years, and it was widespread in patients with coronary heart disease. Uric acid was the final product of purine nucleic acid metabolism in the cell nucleus. When uric acid was excessively produced or excreted in the human body, hyperuricemia will form. Ma et al. [28] believed that UA was an important risk factor for patients with coronary heart disease. Hyperuricemia mainly induced inflammation, damages vascular endothelium, and ultimately activates platelets and coagulation system. At the same time, it improved renin activity, increased platelet adhesion, and promoted thrombosis. It could also cause metabolic abnormalities and has the effect of regulating the formation and metabolism of fat cells. Hyperuricemia was also involved in the body's oxidation and stress and promotes the proliferation of smooth muscle cells. Increased UA levels can promote the oxidation of LDL-C and accelerated the oxidation of lipids. Hyperuricemia had predictive value for the occurrence and development of coronary heart disease.

## 3. Material and Method

### 3.1. Research Object

From September 2018 to March 2019, 290 patients who were admitted to the Department of Cardiology of a third-class hospital in Shanxi who were admitted for suspected or confirmed coronary heart disease and were admitted to the hospital for coronary angiography. Among them, 217 were males and 73 were females, aged 29 to 87 years (average 60.5 ± 9.7 years).

The risk factors included in the analysis included gender, age, hypertension, type 2 diabetes, smoking, blood lipids, uric acid, high-sensitivity C-reactive protein, cystatin C, glycosylated hemoglobin, and fasting blood glucose.

### 3.2. Inclusion and Exclusion Criteria

Inclusion criteria include patients with suspected or diagnosed coronary heart disease at admission and who underwent diagnostic coronary angiography for the first time and who have complete clinical and electrocardiographic data. None of the patients had been treated with lipid-lowering drugs, diuretics, and UA-lowering drugs before hospitalization.

Exclusion criteria include the following: (1) previous interventional therapy; (2) old myocardial infarction; (3) atrial fibrillation; (4) hematological diseases, malignant tumors, or receiving hormone replacement therapy; (5) metabolic diseases; (6) liver and kidney dysfunction; (7) combined with other heart diseases such as rheumatic heart disease; (8) cerebrovascular disease; (9) infectious disease; (10) cardiomyopathy; (11) myocarditis; (12) valvular disease; and (13) clinical data or coronary angiography data are incomplete.

### 3.3. Data Collection

#### 3.3.1. General Data Collection

The electronic medical record management system of the Second Affiliated Hospital of Shantou University Medical College is used to retrieve all patients with suspected or confirmed coronary heart disease and coronary angiography from September 2018 to March 2019. The original medical records were uniformly recalled and checked for all cases, qualified cases were screened in strict accordance with the inclusion and exclusion criteria, and only the first coronary angiography case was selected for repeated admissions to the same patient. The current medical history, past history, family history, smoking history, and physical examination of these eligible patients were collected.

#### 3.3.2. Laboratory Biochemical Index Collection

Biochemical index testing includes uric acid, fasting blood glucose, glycosylated hemoglobin, cystatin C, total cholesterol, triglycerides, high-density lipoprotein, low-density lipoprotein, and high-sensitivity C-reactive protein. The kit company for detecting total cholesterol (TC), triglyceride (TG), high-density lipoprotein, (HDL-C), and low-density lipoprotein cholesterol (LDL-C) is Shanghai Mingdian Bioengineering Co., Ltd. The high-sensitivity C-reactive protein (hs-CRP) kit was provided by Ningbo Kang Biotechnology Co., Ltd. The operation is carried out in strict accordance with the reagent instructions, and the operation is performed by a professional laboratory doctor. The detection and analysis of the above indicators are carried out on the biochemical analyzer of Roche in Germany.

#### 3.3.3. Coronary Angiography

It is performed by a professional cardiologist. The approach is conventional via the femoral artery or radial artery. The left coronary artery is exposed to at least 4 positions, and the right coronary artery is exposed to at least 2 positions. If necessary, other positions are added to the coronary arteries to be fully displayed. For a coronary artery evaluation method, Gensini scoring system [29, 30], according to the different segments of the diseased blood vessel, this scoring formulates different weight coefficients, integrates all coronary artery branches, and calculates the scores of all branches. According to the stenosis score, the degree of stenosis within 25% is counted as 1 point, the degree of stenosis 26%-50% as 2 points, the degree of stenosis 51%-75% as 4 points, the degree of stenosis 76%-90% is counted as 8 points, 91%-99% is counted as 16 points, and completely occluded is counted as 32 points. Multiply the lesion score by the corresponding weight coefficient of the lesion, where the left main stem ×5, the proximal left anterior descending branch ×2.5, the middle ×1.5, the distal and first diagonal branches ×1.0; the proximal left circumflex branch ×2.5, the middle and the distal and posterior descending branches, the proximal, middle, and distal parts of the right coronary artery were all ×1.0; and the small branch ×0.5. The points of each branch were added to obtain the Gensini score of the degree of coronary artery disease in each patient. A Gensini score ≥ 30 points indicates that the patient has 100% coronary artery stenosis and/or multivessel disease. The higher the score, the more obvious the degree of coronary artery disease.

### 3.4. Quality Control

The original medical record verification and related data collection are completed in a unified format. We use Microsoft Excel to establish coronary heart disease and control groups, coronary heart disease groups A and B, and Gensini high and low group databases.

### 3.5. Method of Diagnosis

Coronary heart disease is defined as coronary angiography with one or more main branches of the coronary artery (left main trunk, left anterior descending artery, left circumflex artery, and right coronary artery) vascular diameter stenosis ≥ 50%.

The diagnostic criteria of acute myocardial infarction adopt the global uniform definition of acute myocardial infarction in 2007, and cardiac markers (such as troponin) increase or decrease after increasing. At least one value is greater than 99% of the upper limit of the reference value and has at least one basis for myocardial ischemia: (1) ischemic symptoms, (2) ECG indicates new myocardial ischemia, (3) pathological Q waves, and (4) new myocardial loss or new regional heart wall motion abnormalities.

Hypertension adopts US JNC-VII guidelines: systolic blood pressure (SBP) ≥ 140 mmHg (1 mmHg = 0.133 kPa) and (or) diastolic blood pressure (DBP) ≥ 90 mmHg in resting state twice, or have a clear history of hypertension, except for secondary hypertension.

The diagnostic criteria for type 2 diabetes are based on the 2014 American Diabetes Association standard: fasting blood glucose ≥ 7 mmol/L (126 mg/dL), or glucose tolerance test 2-hour blood glucose ≥ 11.1 mmol/L (200 mg/dL).

Smoking is defined as smoking at least 1 cigarette a day, and smoking continuously for more than 1 year, still smoking now or quitting smoking less than half a year when enrolled in this study. Those who quit smoking for more than half a year are listed as nonsmokers.

Dyslipidemia is defined as cholesterol (TC) ≥ 5.72 mmol/L (200 mg/dL) and (or) triglyceride (TG) ≥ 1.70 mmol/L (150 mg/dL) and (or) high‐density lipoprotein cholesterol (HDL‐C) < 1.04 mmol/L (40 mg/dL), and (or) low‐density lipoprotein cholesterol (LDL‐C) ≥ 3.64 mmol/L (140 mg/dL).

Hyperuricemia is defined as blood uric acid levels in men > 420 *μ*mol/L (7 mg/dL) and women > 375 *μ*mol/L (6 mg/dL).

### 3.6. Grouping Principle

According to the results of coronary angiography, patients with coronary artery stenosis ≥ 50% (*n* = 202) were regarded as the coronary heart disease group, and patients with coronary artery stenosis < 50% were regarded as the control group (*n* = 88). In the coronary heart disease group, patients with acute myocardial infarction were regarded as coronary heart disease group A (*n* = 109), and patients with coronary heart disease except acute myocardial infarction were regarded as coronary heart disease group B (*n* = 93). According to the results of the Gensini score, patients with scores less than 30 are classified as the Gensini low group (*n* = 157), and patients with scores greater than or equal to 30 are classified as the Gensini high group (*n* = 133).

### 3.7. Computer-Aided Statistical Method

All data were statistically analyzed using SPSS22.0 software (IBM, Armonk, NY, USA). Measurement data were expressed as mean ± standard deviation (*x* ± *s*), and independent sample *t*-test was used for comparison between the two groups. The skewness data is expressed by the median and interquartile range, and the rank sum test is used for comparison between the two groups. Enumeration data is expressed by composition ratio, and the comparison of the composition ratio of two samples is performed by chi-square test. The correlation between coronary heart disease risk factors and Gensini score was analyzed by Spearman correlation analysis, and the correlation between the two after controlling for interference factors was compared using partial correlation analysis; the relationship between coronary heart disease risk factors and Gensini score was analyzed by multiple linear regression analysis. The relationship between the risk factors of coronary heart disease and the risk of coronary heart disease was analyzed by binary logistic regression. *P* < 0.05 indicates that the difference is statistically significant, and *P* < 0.01 indicates that the difference is significant.

## 4. Experiment

### 4.1. Comparison of Basic Data between CHD Group and Control Group

A total of 290 qualified cases were collected, including 202 cases in the coronary heart disease group and 88 cases in the control group. The risk factors that conform to the normal distribution in the measurement data are age, UA, and LDL-C, expressed as mean ± standard deviation (*x* ± *s*), and independent sample *t*-test is used for comparison between the two groups. The risk factors with skewed distribution in the measurement data are FBG, HbA1c, HDL-C, CysC, TC, TG, and hs-CRP, expressed in median and interquartile range, and the rank sum test was used for comparison between the two groups. The count data included gender, history of hypertension, history of diabetes, and history of smoking, expressed as a constituent ratio, and the chi-square test was used for comparison between the two groups.

Chi-square analysis (Table 1 and Figure 2) shows that the proportion of men in coronary heart disease and the control group is higher than that of women, and the proportion of hypertension, diabetes and smoking history is significantly higher than that in the control group. The difference is statistically significant (*P* < 0.01). In the two independent sample *t*-tests (Table 2 and Figure 3). The levels of UA and LDL-C were higher than those of the control group, and the difference was statistically significant (*P* < 0.05). The rank sum test (Figure 4) found that there was no statistically significant difference between FBG and CysC between the control group and the coronary heart disease group (*P* > 0.05). The medians between the HDL-C groups were, respectively, 1.2 and 1.0, and the difference is statistically significant (*P* < 0.05).

### 4.2. Comparison of Basic Data of CHD-A and CHD-B

The diagnostic criteria for acute myocardial infarction adopt the 2007 global unified definition of acute myocardial infarction. The patients with acute myocardial infarction in the coronary heart disease group were regarded as the coronary heart disease group A (*n* = 109), and the patients with coronary heart disease except acute myocardial infarction were regarded as the coronary heart disease group B (*n* = 93). Measurement data conforming to the normal distribution include age, UA, and LDL-C, expressed as mean ± standard deviation (*x* ± *s*), and the independent sample *t*-test is used for comparison. The measurement data that does not conform to the normal distribution include HbA1c, TC, TG, HDL-C, and hs-CRP, which are expressed in median and interquartile range, and the rank sum test is used for comparison. The count data included gender, history of hypertension, history of diabetes, and history of smoking, expressed as a constituent ratio, and the chi-square test was used for comparison. In the measurement data (Table 3 and Figure 5), gender, history of hypertension, history of diabetes, and history of smoking were not statistically significant between groups A and B of coronary heart disease. The *t*-test of two independent samples (Table 4) showed that the age of onset of group A was smaller than that of group B, and the UA level was significantly lower than that of group B (*P* < 0.01), the difference was statistically significant (*P* < 0.05), LDL-C. The comparison between the two groups was not statistically significant. In the rank sum test (Table 5 and Figure 6), the difference between the two groups of hs-CRP was statistically significant (*P* < 0.01), and the remaining risk factors were not statistically significant between group A and group B as shown in Table 6 (*P* > 0.05).

### 4.3. Correlation Analysis of Risk Factors and Gensini Score

Spearman correlation analysis (Table 7) shows that the risk factors of TG, LDL-C, and hs-CRP in patients with coronary heart disease are positively correlated with the degree of coronary heart disease stenosis (*r* > 0, *P* < 0.05), while HDL-C is associated with coronary heart disease. The degree of heart disease stenosis was negatively correlated (*r* < 0, *P* < 0.05). However, after adjusting for factors such as gender, hypertension, diabetes, and smoking, partial correlation analysis (Table 8) found that hs-CRP is still closely related to Gensini score, and the difference is statistically significant (*r* = 0.2, *P* = 0.009). However, the correlation between other risk factors and Gensini score was not statistically significant (*P* > 0.05).

### 4.4. Regression Analysis of Relationship between Risk Factors and Gensini Score

With the Gensini score of coronary heart disease as the dependent variable and the risk factors of coronary heart disease as the independent variable, the independent variable entry method used stepwise entry, and multiple linear regression analysis was performed (Table 9). The results showed that the partial regression coefficients of smoking history, diabetes history, hs-CRP, age, and low-density lipoprotein and Gensini score were statistically significant (*P* < 0.05), and the remaining risk factors were not statistically significant with Gensini score (*P* > 0.05).

### 4.5. Logistic Analysis of Relationship between Risk Factors and Outcomes

We dichotomize UA, FBG, HbA1c, CysC, TC, TG, HDL-C, LDL-C, hs-CRP by median. We define the higher quantile group as the high quantile group and define the lower quantile group as the lower quantile group. With coronary heart disease as the dependent variable and coronary heart disease risk factors as the independent variable, the independent variable entry method uses the forward LR method, and the binary logistic regression analysis is performed. Binary logistic regression analysis (Table 10) found that age, smoking history, hs-CRP, and HbA1c can be used as a risk factor for predicting coronary heart disease (*P* < 0.05). The partial regression coefficient *B* of age is 0.043, the OR value is 1.04, *P* < 0.05, which is statistically significant, for the high hs-CRP group and high HbA1c group. Compared with the low quantile group, the risk of coronary heart disease was significantly higher, and the difference was statistically significant. The risk of coronary heart disease among smokers was 4.894 times higher than that of nonsmokers, and the difference was statistically significant. The other independent variables were not statistically significant compared with the control group.

## 5. Discussion

This study excluded previous interventional therapy, old myocardial infarction, atrial fibrillation, hematological diseases, malignant tumors or receiving hormone replacement therapy, metabolic diseases, liver and kidney insufficiency, and other heart diseases such as rheumatic heart disease., cerebrovascular disease, infectious disease, cardiomyopathy, myocarditis, and valvular disease. It was found that patients with coronary heart disease were older than the control group (*P* < 0.05), the proportion of men was higher than that of women, and the proportion of hypertension, diabetes, and smoking was significantly higher than that of the control group (*P* < 0.01). It is basically the same as the previous literature. It suggests that age, sex, hypertension, diabetes, and smoking are importantly related to the onset of coronary heart disease and may be involved in the formation of coronary heart disease.

In multiple linear regression, the partial regression coefficients of smoking, diabetes, and Gensini score are statistically significant, suggesting that smoking and diabetes are important risk factors for coronary heart disease, and both have an important relationship with the degree of coronary artery stenosis in patients with coronary heart disease. It is considered that smoking causes damage to the endothelium of arteries and leads to a decline in endothelial-dependent diastolic function. The long-term hyperglycemia state causes lipid metabolism disorders, the level of cardioprotective HDL-C decreases and LDL-C increases, LDL-C is easily oxidized, and the end products of glycosylation reduce the compliance of the arterial wall. All of the above can aggravate the degree of atherosclerosis. Binary logistic regression analysis found that the older the age, the greater the risk of coronary heart disease. The risk of coronary heart disease in smokers was 4.894 times that of nonsmokers. The difference was statistically significant, suggesting that age and smoking are independent risk factors for coronary heart disease.

This study also found that UA, hs-CRP, HbA1c, TC, TG, and LDL-C in patients with coronary heart disease were higher than those in the control group, while HDL-C was relatively low, and the difference was statistically significant (*P* < 0.05). FBG and CysC were not statistically significant between the two groups (*P* < 0.05). It is suggested that UA, hs-CRP, HbA1c, and hyperlipidemia may be involved in the pathogenesis of coronary heart disease as risk factors for coronary heart disease. Increased HDL-C is a protective factor for coronary heart disease and plays a protective effect on the heart. However, FBG and CysC may not be involved in the formation of coronary heart disease.

It can be seen from the multiple linear regression analysis that the partial regression coefficients of hs-CRP and LDL-C and Gensini scores are statistically significant when multiple risk factors are involved. It is suggested that after considering multiple factors, hs-CRP and LDL-C are still closely related to the degree of coronary artery stenosis. The higher the level of hs-CRP and LDL-C, the greater the degree of coronary artery stenosis. Consider that during the onset of coronary heart disease, the increase in hs-CRP may be secondary to the activation of the complement system and the release of inflammatory mediators, causing hyperplasia of the coagulation-fibrinolysis system after vascular intimal damage, platelet aggregation, and thrombosis, leading to aggravation of coronary artery stenosis. Increased levels of LDL-C will deposit in the arterial wall, gradually forming atherosclerotic plaques, blocking blood vessels, and aggravating the severity of coronary heart disease. Binary logistic regression analysis found that the risk of coronary heart disease increased by 8.923 times in the high-hs-CRP group compared with the low-hs-CRP group; the risk of coronary heart disease increased by 2.992 times in the high-HbA1c group compared with the low-HbA1c group. It was statistically significant (*P* < 0.05), indicating that hs-CRP and HbA1c are independent risk factors for coronary heart disease. The higher the level of hs-CRP and HbA1c, the greater the risk of coronary heart disease. Among them, high hs-CRP is the most significant risk factor for coronary heart disease among independent risk factors.

Comparing coronary heart disease group A with group B, it can be seen that the age of patients with acute myocardial infarction is slightly lower than that of other patients with coronary heart disease except acute myocardial infarction (*P* = 0.046), but the difference between the two groups is not very significant. The level of hs-CRP in patients with acute myocardial infarction was significantly higher than that in patients with coronary heart disease without acute myocardial infarction (*P* < 0.01), and the difference was statistically significant, suggesting that hs-CRP may represent one of the indicators of acute exacerbation of coronary heart disease. The level of uric acid UA in coronary heart disease is higher than that in the control group. However, in patients with acute myocardial infarction, it is significantly lower than that in patients with nonacute myocardial infarction. It is not excluded that the number of cases in our study population is small, and the results are biased and need to be further explored in the future. The levels of HbA1c, TC, TG, and LDL-C in coronary heart disease group A were slightly lower than those of group B, and HDL-C was slightly higher than that of group B, but there was no statistically significant difference between the two groups (*P* > 0.05). It is suggested that gender; hypertension; diabetes; smoking; increased HbA1c, TC, TG, and LDL-C; and decreased HDL-C may not be the key factors of acute coronary heart disease.

This study found that the age, gender, hypertension, diabetes prevalence, and smoking composition ratio, UA, HDL-C, LDL-C, HbA1c, TC, TG, and hs-CRP of patients with coronary heart disease are different from those of the control group. It was statistically significant, suggesting that rising age, males, hypertension, diabetes, smoking, hyperuricemia, dyslipidemia, and high hs-CRP are involved in the formation of coronary heart disease, while the comparison between FBG and CysC is not statistically significant. It suggests that the two may not be important factors in the occurrence and development of coronary heart disease.

In this study, a single factor correlation analysis found that hs-CRP in patients with coronary heart disease showed an increasing trend with the severity of coronary artery disease. After adjusting for gender, hypertension, diabetes, and smoking, hs-CRP was still correlated with the degree of coronary heart disease stenosis. It was positively correlated, and the difference was statistically significant (*P* < 0.05). At the same time, through multivariate correlation analysis, the partial regression coefficients of hs-CRP and Gensini scores were statistically significant, suggesting that hs-CRP is the most correlated degree of coronary artery stenosis. Controlling risk factors may play an important role in causing further coronary artery stenosis. Further binary logistic regression analysis showed that hs-CRP also showed a high correlation, suggesting that high-sensitivity C-reactive protein has a predictive effect on the likelihood of coronary heart disease, and relevant attention needs to be drawn.

In this study, through binary logistic regression analysis, it was found that the higher the glycosylated hemoglobin in patients with coronary heart disease, the higher the risk of coronary heart disease, suggesting that elevated glycosylated hemoglobin can also be used as one of the early warning factors for predicting coronary heart disease.

## 6. Conclusion

Old age, men, hypertension, diabetes, smoking, hyperuricemia, dyslipidemia, and high hs-CRP may be involved in the occurrence and development of coronary heart disease. And age, smoking, hs-CRP, and HbA1c are independent risk factors for coronary heart disease. Among them, hs-CRP predicts coronary heart disease with higher value than HbA1c, smoking history and age. Age, UA, and hs-CRP may be involved in the process of acute coronary heart disease. Men, hypertension, diabetes, smoking, decreased HDL-C, increased LDL-C, TG, and hs-CRP may be involved in the development of the severity of coronary artery disease. Among them, hs-CRP is the most relevant risk factor for the degree of coronary artery stenosis, and may play an important role in causing further coronary artery stenosis. In summary, among the risk factors for coronary heart disease, age, smoking, hs-CRP, and HbA1c are independent risk factors for coronary heart disease, and hs-CRP is the most significant controllable independent risk factor for coronary heart disease. By controlling smoking, reducing the levels of glycosylated hemoglobin and hs-CRP, preventing diabetes and controlling inflammation may be one of the measures to control the aggravation of coronary artery stenosis in coronary heart disease.

## Figures and Tables

**Figure 1:** The cardiovascular disease.

**Figure 2:** Comparison of basic data between the CHD group and control group.

**Figure 3:** Comparison of basic data between the CHD group and control group.

**Figure 4:** Comparison of basic data between the CHD group and control group.

**Figure 5:** Comparison of basic data between CHD-A and CHD-B.

**Figure 6:** Comparison of basic data between CHD-A and CHD-B.

**Table 1:** Comparison of basic data between the CHD group and control group.

Item	*χ* ^2^	*P*
Male	5.9	0.013
Hypertension	5.6	0.017
Diabetes	7.2	0.007
Smoking	13.7	0.001

**Table 2:** Comparison of basic data between the CHD group and control group.

Item	*t*	*P*
Age	2.6	0.022
UA	2.9	0.043
LDL-C	1.8	0.034

**Table 3:** Comparison of basic data between CHD-A and CHD-B.

Item	*χ* ^2^	*P*
Male	0.9	0.439
Hypertension	0.1	0.951
Diabetes	1.7	0.175
Smoking	0.7	0.429

**Table 4:** Comparison of basic data between CHD-A and CHD-B.

Item	*t*	*P*
Age	-2.7	0.041
UA	-3.4	0.019
LDL-C	-0.9	0.533

**Table 5:** Comparison of basic data between CHD-A and CHD-B.

Item	*T*	*P*
HbA1c	5753.7	0.849
TC	8765.7	0.448
TG	10855.2	0.602
HDL-C	9192.3	0.554
hs-CRP	6783.2	0.000

**Table 6:** Spearman correlation analysis of risk factors and Gensini score.

Item	Gensini score	
	*r*	*P*
TG	0.14	0.015
HDL-C	-0.20	0.001
LDL-C	0.13	0.023
hs-CRP	0.42	0.000

**Table 7:** Analysis of partial correlation between risk factors and Gensini score.

Item	Gensini score	
	*r*	*P*
TG	0.06	0.416
HDL-C	-0.04	0.515
LDL-C	0.13	0.052
hs-CRP	0.18	0.009

**Table 8:** Multiple linear regression analysis of risk factors and Gensini score.

Item	*B* (95% CI)	SB	*P*
hs-CRP	0.29 (0.83~ 0.49)	0.18	0.006
Smoking	18.60 (8.83~ 28.36)	0.25	0.000
Diabetes	11.81 (2.18~ 21.45)	0.16	0.016
LDL-C	5.20 (0.13~ 10.28)	0.13	0.045

**Table 9:** Two-class logistic regression analysis of risk factors.

Item	*B* ± SE	OR (95% CI)	*P*
Age	0.04 ± 0.02	1.04	0.025
Smoking	1.59 ± 0.37	4.89	0.000
High HbA1c	1.10 ± 0.37	2.99	0.003
High Hs-CRP	2.19 ± 0.39	8.92	0.000

## Data Availability

The data underlying the results presented in the study are available within the manuscript.
